# Application of Magnetic Resonance Imaging of Patients with Concussion in Clinical Emergency

**DOI:** 10.1155/2021/7749540

**Published:** 2021-12-01

**Authors:** Peng Fang, Dezhao Lin, Ka Xu, Shangyan Ying

**Affiliations:** Wenzhou Hospital of Tradition Chinese Medicine, Wenzhou, Zhejiang, China 325000

## Abstract

Concussion syndrome is a common disease in neurosurgery, and its incidence ranks first among all traumatic brain injuries. Cognitive dysfunction is one of the most common functional impairments in concussion syndrome. Neuroimaging and content assessments on concussion patients and healthy control subjects are used in this study, which uses MRI technology to evaluate brain pictures of concussion patients. Moreover, this paper separately evaluates the scores of the concussion syndrome group and the healthy control group in multiple functional aspects and performs independent sample *t*-test after statistics of the two scores. In addition, this paper uses resting-state fMRI to study the changes in the functional connectivity of the medial prefrontal lobe in patients with PCS, which has certain significance in revealing cognitive dysfunction after concussion and has a certain effect on improving the clinical emergency diagnosis and treatment of concussion.

## 1. Introduction

The most prevalent kind of head injury is concussion. However, today's concussion diagnosis is still dependent on the patient's medical history and symptoms, as well as the receiving physician's medical opinion. Furthermore, there is a lack of clear pathophysiological mechanisms as well as objective and clear imaging evidence to confirm the diagnosis, and there is still a lack of consensus on diagnosis and treatment guidelines, resulting in differences in clinical diagnosis and the diagnosis of concussion becoming the subject of judicial controversy [1]. Most previous perspectives held that neurological dysfunction after a concussion had no obvious neuroanatomical foundation, that cognitive issues may be the primary mechanism of PCS, and that emotional and psychological factors play a significant role in symptom maintenance. Furthermore, there is presently no especially effective therapy for concussion syndrome, and the primary treatment is symptomatic and supportive care, which has an unreliable impact. As a result, concussion syndrome has a significant impact on patients' daily lives and jobs, resulting in significant waste of medical resources and family hardship, as well as a negative impact on society's economy. Patients with a concussion need to be evaluated using trustworthy and precise laboratory indicators to properly pinpoint their brain damage location and assess their level of injury, so that the injury and prognosis may be reliably determined. Moreover, it can provide a reliable basis for clear clinical diagnosis, timely treatment, and judicial appraisal. At the same time, studying the brain function of concussion patients during the recovery period will help to understand the neural mechanism of concussion syndrome. Traumatic brain injury causes shear strain to be created at the junction, which causes damage to the cell membrane, axons, and the brain's blood vessels as a result of the varied densities of brain tissue in various sections of the brain [2]. After the integrity of the nerve cell membrane and the destruction of the blood-brain barrier, the ion channels are opened to cause the release of related excitatory neurotransmitters such as acetylcholine and potassium ions to increase [3]. At this time, the destruction of the blood-brain barrier, changes in cerebral blood flow, rupture of lysosomal membranes, and the number of neuronal cells can all be affected [4]. This is the pathological mechanism why patients with concussion syndrome continue to have headaches, dizziness, memory impairment, and cognitive impairment. Attention, executive function, memory, and high-level abstract thinking are only few of the high-level capabilities specific to the human brain that play a vital part in the processing of information that is received. In addition, studies have found that in addition to the long-term selective attention disorder in PCS patients, attention disorder may also exist for a long time.

On the basis of MRI technology, brain functional magnetic resonance imaging technology has been created. Since blood oxygen level-dependent fMRI (BLOD-fMRI) has been used for magnetic resonance brain functional imaging technology, it has been discovered that it has good space, time resolution, fast imaging speed, no radiation, easy positioning, noninvasive approach, strong reproducibility, and other advantages. The benefits have been swiftly expanded, and it is now extensively employed in the study of cranial nerve function, neuropsychological function, and other popular disciplines. The shape and function of brain tissue, as well as its connections, provide a novel perspective. The imaging premise of BOLD-fMRI is that when neuronal cell activity increases, so does local cerebral blood flow and oxygen consumption; however, owing to asynchrony, the rise in oxygen consumption is slower than the increase in cerebral blood flow. When compared to the resting state, the active brain region's venous blood oxygen content is much greater than the surrounding inactive area tissue, resulting in a comparatively enhanced local brain tissue signal on T2-weighted functional magnetic resonance imaging. Traditional imaging technologies that have been utilized in the past, such as positron emission tomography (PET), need imaging and display and depend on the change in blood oxygen content in the body as a natural contrast agent; imaging indicates changes in brain tissue microscopically. BOLD-fMRI is a noninvasive and nonradiation approach that gives excellent temporal and spatial resolution. As a result, it has been extensively employed in brain function research in recent years. Some researchers studied concussion syndrome using BOLD-fMRI function connection, brain network properties, DTI (diffusion tensor imaging), magnetoencephalogram, and other approaches and discovered that individuals with concussion syndrome had abnormal brain function and microbrain tissue structure. It is obvious that something is wrong.

This research examines the use of MRI in the clinical emergency of patients with concussion, aiming to enhance the diagnosis and treatment of emergency concussion patients while lowering their clinical risk.

## 2. Related Work

Due to the different densities of brain tissue in different parts, when brain trauma occurs, the shear force generated at the junction will cause pathological changes such as cerebral cortex tissue contusion, cell membrane destruction, microvascular injury, and progressive traction injury of the axons [5]. When metabolism is disordered, brain metabolism, cell function, blood-brain barrier, etc. are all affected. This may be the cause of persistent headache, dizziness, memory impairment, cognitive impairment, and other manifestations in patients with postconcussion syndrome. The previous view held that there is no substantial damage to the brain tissue after a concussion, but only due to individual psychological factors. However, existing scholars have found that S100B protein changes may have a certain correlation with patients' cognitive dysfunction [6]. Cognitive function belongs to the high-level functions unique to the human brain, mainly including attention, executive function, memory, and high-level abstract thinking [7]. Studies have found that a large part of mTBI patients have varying degrees of attention deficit after injury, and attention deficit persists for a long time after injury. The brain tissue has a localized nerve fiber bundle structural disorder, which manifests as nerve fiber bundle rupture disorder and focal axonal membrane injury, according to related study on the structure of concussion [8]. According to the literature [9], high-precision fiber tracking technology identified rupture and destruction of nerve fiber bundles, impairment to the integrity of the blood-brain barrier, and alterations in brain permeability in patients with moderate head injuries who had no major complaints or bothersome symptoms. The activity of local brain regions was dramatically decreased when PET was used to analyze individuals with postconcussion syndrome.

Clinical cognitive dysfunction evaluation measures include the Glasgow Coma Scale, Memory Forgetting Test, Galveston Orientation Test Scale, and Montreal Cognitive Assessment Scale. The patient's postinjury awareness (eye-opening activity, bodily movement, and response language), orientation, memory, and cognition are all evaluated using these measures [10]. Glasgow Coma Scale scores show a strong association with MoCA and GOAT scores, according to clinical experience and a significant number of follow-up research. Through the assessment of the patients' self-reported symptoms, they were divided into three grades: mild, moderate, and severe, according to the scores after the assessment. Finally, the severity is classified according to the total score. This is the evaluation principle of the postconcussion symptom scale (PCSS) and the Rivermead concussion sequela questionnaire. The level of cognitive impairment following a concussion may be determined by the difference in the final total score. A vast number of clinical analytic investigations have proven that both PCSS and RPQ have strong test-retest reliability and surface structure validity at this time [11]. Some scholars use functional MRI to evaluate the effectiveness of concussion syndrome and found that the concussion sequela score is negatively correlated with the cognitive evaluation subscale score. This conclusion supports the use of self-evaluated PCSS scores to diagnose and evaluate mTBI cognitive dysfunction and its rehabilitation [12].

Functional magnetic resonance imaging (fMRI) is a new type of magnetic resonance imaging technology. It uses the oxygen level-dependent (BOID) technology to detect changes in brain metabolism, that is, to detect the BOLD signal, and use the internal relationship between brain oxygen consumption and brain function to complete the evaluation of brain function. CT or conventional MRI in most patients with concussion are normal, but they continue to show related cognitive dysfunction. The use of functional magnetic resonance technology to collect and analyze relevant data in patients with concussion can detect functional abnormalities and structural network damage between the internal functional areas of the brain at an early stage. It offers a precise imaging foundation for the diagnosis and treatment of postconcussion illness since it can gather functional connection data of the sequelae of mTBI [13]. When researching the neural basis of memory impairment in patients with concussion, the literature [14] revealed that event-related fMRI is extremely sensitive to the directional diagnosis of patients with mild brain damage. The ongoing cognitive impairment of troops following battle injuries was studied using fMRI in the literature [15]. The concussion patient group revealed activation in associated brain regions such as the anterior and posterior cingulate gyrus, the medial prefrontal lobe, and the parietal lobe, as well as apparent abnormalities in various brain locations. This might be the neurological process causing the wounded person's cognitive impairment. The resting-state functional connectivity of the thalamus cortex in patients with concussion syndrome was dramatically improved by the resting-state MR investigation, according to the literature [16]. The resting-state functional magnetic resonance seed point functional connection method was used in the literature [17] to study postmemory impairment in patients with mTBI and found that the memory impairment is caused by a weakened functional connection between the parahippocampal gyrus and various brain regions throughout the whole brain. It investigates memory impairment in individuals with mTBI using the functional connection approach in fMRI. The functional relationship between the parahippocampal gyrus and the bilateral prefrontal lobes, temporal lobes, and other areas of mTBI patients was shown to be decreased, which explained the alterations in memory loss and cognitive impairment following mTBI.

## 3. Materials and Methods

We initially include relevant eligible patients based on the diagnostic criteria for concussion in DSM-IV and collect relevant patient data in the hospital. The criteria for inclusion in the experimental patient group are as follows: (1) the patient has a clear history of traumatic brain injury, and the Glasgow Coma Score (GCS) is between 13 and 15 points. Moreover, the patient has a short-term disturbance of consciousness after the trauma, and the disturbance of consciousness lasts for several minutes, but the coma is within half an hour, the amnesia after the trauma does not exceed 24 hours, and the change of consciousness and mental state does not exceed 24 hours; (2) the patient has a series of related clinical symptoms after injury: such as headache, dizziness, nausea and vomiting, tinnitus, insomnia, photophobia, decreased concentration, irritability, and fatigue. Sluggishness, difficulties with short- and long-term memory, sleep disturbances, inability to focus, and other conscious symptoms are also reported by patients, and the symptoms are chronic, recurrent, or persistent and cannot be eased; (3) the patient who still has symptoms of concussion syndrome 3 months after the event; and (4) the patients' regular neuroimaging scans revealed no positive findings such as fractures, intracerebral hematomas, or diffuse axonal damage. At the same time, our research group recruit 27 healthy volunteers as the control experimental group, set the relevant inclusion conditions, and matched the age, gender, and education level. The selection and inclusion criteria of the concussion syndrome patient group and healthy control group with cognitive dysfunction are as follows: (1) right-handed; (2) no serious physical disability or disease such as heart, liver, and kidney disease; (3) no history of mental disorders, learning disabilities, attention deficit disorders, and other neurological and psychiatric diseases; (4) first-degree relatives have no history of neuropsychiatric disease; (5) no claustrophobic syndrome, foreign body implantation, and other contraindications for MRI examination; (6) no history of addiction or abuse of toxic substances, alcohol, and psychotropic drugs; and (6) no history of traumatic brain injury, and there is no obvious substantive disease on conventional cranial CT and MRI scans. The experiment is based on the principle of voluntariness. It informs the purpose of the experiment, the experiment process, and the related obligations and rights. After obtaining the consent of the volunteers, the informed consent form is signed and submitted to the school and the hospital ethics committee for approval [18].

We use MoCA to test the following content in the concussion syndrome group and the healthy control group: 6 content tests including naming, attention, abstraction, words, visual space executive function, and delayed memory. The results of the concussion syndrome group and the healthy control group are compared in terms of name, attention, abstraction, vocabulary, visual spatial executive function, delayed memory, and so on, and the independent sample *t*-test is used after the two groups' total scores have been tallied.

After obtaining the DICOM format data, we first use the MRIConvert software to convert the data to the NIFTI format and then preprocess the experimentally obtained images through the SPM8 software package. The first 10 image data of each subject may cause errors due to factors such as the instability of the machine and the subject, so they are eliminated during preprocessing, and only the remaining 170 reliable dynamics are preprocessed.

The subjects were warned ahead of time to keep their heads still, and their heads were also appropriately secured. In the course of gathering data, however, a minor head shake is inevitable. Due to the extreme sensitivity of magnetic resonance imaging, even the tiniest movement may interfere with proper imaging, leading the pixel correspondence across multiple scans to be lost. As a result, each picture frame acquired from the experiment is aligned with the first image frame in this TR. To correct each subject's head movement, we employ the rigid body model's spatial transformation with 6 parameters (translation in the three dimensions of *x*, *y*, and *z*) and rotation in these three directions. Furthermore, data having a rotation of more than 1.5 degrees and a translation of more than 1.5 mm is usually excluded. This experiment's data collecting proceeded easily, and the analysis revealed that no data from the participants needed to be removed.

Not all pictures are scanned at the same time in the fMRI data capture and scanning process, and there is a tiny time gap between each layer of scanning. The BOLD signal will vary even if there is a little variation. The BOLD signal obtained by neighbouring pictures will be affected by the time difference in real scanning. As a result, we conduct time correction on the data of each layer acquired in each TR to ensure that the image acquisition time of each layer in a TR is constant, reducing the influence of the time difference between layers on data processing. That is, all of the photos captured at the same moment are scanned simultaneously [19].

The picture is smoothed using the Gaussian smoothing function to make the image data more compatible with the Gaussian field distribution and to eliminate disparities in brain sulcus and gyrus structure across different participants and to boost the signal-to-noise ratio (SNR) (normal distribution). To conduct spatial smoothing on the experimental photos, a Gaussian smoothing check with a full width at half maximum (FWHM) value of 4 mm was utilized. Low-frequency signal drift and high-frequency noise, such as breathing and pulse, were reduced in order to improve the experimental outcomes. The processed data is subjected to low-frequency filtering (0.01 Hz~0.08 Hz), linear drift processing, and other reprocessing. Moreover, the experimental error signal caused by the patient's head movement and the cerebrospinal fluid signal and white matter signal in the brain itself are removed, so that the experimental results are more reliable and a 90 × 90 matrix with AAL_90 as the template is established [20].

## 4. Result

By analyzing the general conditions of the PCS group (patient group) and HC group members such as gender, age, and educational level, we found that the difference was not statistically significant, as shown in Table 1.

WM used MoCA to evaluate the concussion syndrome group and the healthy control group and analyze the results. The results show that the difference in MoCA scores between the PCS group and the HC group is statistically significant. The results are shown in Tables 2–7.

We use the left medial prefrontal lobe as the ROI for functional connectivity analysis. Compared with the HC group, the brain areas in the PCS group with weakened functional connection to the left medial prefrontal lobe include the bilateral lenticular nucleus, left subfrontal gyrus, left insula, right subfrontal gyrus, superior frontal gyrus, middle frontal gyrus, inferior frontal gyrus, and right middle temporal gyrus. However, the functional connectivity of the left fusiform gyrus, left middle temporal gyrus, left superior temporal gyrus, and left superior lobule show enhancement (*P* < 0.05) (Table 8). We use the right medial prefrontal cortex as the ROI for functional connectivity analysis. The PCS group's brain areas showing weakened functional connectivity are the bilateral inferior parietal lobules, left central anterior gyrus, right central posterior gyrus, and talus. The functional connection between the right inferior temporal gyrus and the left parahippocampal gyrus was enhanced (*P* < 0.05) (Table 9). The PCS group and the HC group had a statistically significant difference in the results of functional connection analysis (*P* < 0.05).

## 5. Conclusion

The ROI for this investigation was the left and right medial prefrontal lobes, which were utilized to calculate functional connections throughout the whole brain. The ROI for the functional link investigation was the left medial prefrontal lobe. The concussion syndrome group was compared to the healthy control group in the left medial prefrontal lobe. The left putamen, left insula, right putamen, right middle temporal gyrus, left subfrontal gyrus, upper frontal gyrus, and middle frontal gyrus are the brain locations with impaired cortical functional connections. Functional connectivity has improved in the left superior temporal gyrus, left middle temporal gyrus, left superior lobule, and left fusiform gyrus; the right medial prefrontal lobe is used as the ROI for functional connectivity analysis, suggesting PCS. Functional connectivity was reduced in the bilateral inferior parietal lobules, left central anterior gyrus, right central posterior gyrus, and talus gyrus; functional connectivity was enhanced in the right inferior temporal gyrus and left parahippocampal gyrus. The outcomes of these studies should help researchers figure out what causes cognitive decline following a concussion: (1) the default network includes the medial prefrontal cortex, the inferior parietal lobule, and the angular gyrus of the inferior parietal lobule. A recent study has connected the default network to cognitive decline. The inferior lobules constitute the vigilant attention network, and most of these brain areas are active under calm settings. They play a critical role in executive function, spatial orientation, and memory. The inferior lobe, as the cortical sensory centre of the brain, controls the human body's complex sensations, body image disorders, dyslexia, and apraxia and is related to mathematics and logic; and the superior lobe, as the cortical sensory centre of the brain, participates in the attention target positioning function of visual space related information; and the superior lobe, as the cortical sensory centre of the brain, controls the human body's complex sensations and dyslexia. Capabilities are linked to aspects. The functional relationship between the inferior parietal lobule and the medial prefrontal lobe seems to be decreased in this research, which might explain cognitive anomalies such as attention, complex sensation, body image disorder, dyslexia, apraxia, and memory impairment. In this experiment, the medial prefrontal cortex, the brain's frontal cortex, and the temporal cortex are all significantly weakened, resulting in a decrease in information exchange between the central cortex and the medial prefrontal cortex, which obstructs the processing of various cognitive information. It might be the source of cognitive impairment after a concussion. Moreover, this study showed that the functional connection between the medial prefrontal cortex and the bilateral parahippocampal gyrus was enhanced. It may be a compensatory mechanism of the body. The parahippocampal gyrus strengthens the functional connection with the frontal lobe, improves the efficiency of episodic memory processing, and may alleviate the symptoms of memory decline.

This study shows that the functional connection between the medial prefrontal lobe and the central anterior gyrus and central posterior gyrus is weakened, which may be related to the processing and transmission of primary sensory and motor information. The specific mechanism remains to be further studied. This study uses resting-state fMRI to study the changes in the functional connectivity of the medial prefrontal lobe in patients with PCS, which has a certain significance in revealing the cognitive dysfunction after a concussion. The next step is to conduct a more in-depth study on the relationship between specific functional injury sites to further reveal the neural mechanism of PCS.

## Figures and Tables

**Table 1:** Gender, age, and education level of the test group and control group.

Project	*t* value/*χ*^2^ value	*P* value
Gender of cases (male/female)	0.211	0.643
Age (years old)	0.817	0.187
Education level (years)	1.321	0.079

**Table 2:** Comparison of the naming test between the experimental group and the control group.

Number	PCS group	Control group	Number	PCS group	Control group	Number	PCS group	Control group
1	2.03	3.19	13	2.14	2.88	25	2.40	3.21
2	2.35	2.88	14	2.22	3.18	26	2.64	2.70
3	2.48	2.97	15	2.50	2.76	27	2.01	2.66
4	2.53	2.75	16	2.04	2.93	28	2.63	2.77
5	2.42	3.09	17	2.05	2.67	29	2.62	2.72
6	2.34	2.85	18	1.90	3.28	30	2.11	2.86
7	2.21	3.26	19	2.04	2.69	31	2.53	2.86
8	2.46	3.09	20	2.19	2.88	32	2.24	2.77
9	2.02	2.99	21	2.64	3.30	33	2.54	2.99
10	2.04	3.03	22	2.32	3.27	34	2.24	2.79
11	2.53	3.03	23	2.42	3.00	35	2.60	2.88
12	2.61	3.18	24	1.95	2.90	36	2.04	2.73

**Table 3:** Comparison of the attention test between the experimental group and the control group.

Number	PCS group	Control group	Number	PCS group	Control group	Number	PCS group	Control group
1	2.54	2.64	13	2.60	2.72	25	2.55	2.67
2	2.49	3.11	14	2.70	2.44	26	2.64	3.11
3	2.71	2.75	15	2.44	2.42	27	2.47	2.37
4	2.66	3.00	16	2.30	3.18	28	2.64	2.55
5	2.28	2.56	17	2.28	2.36	29	2.72	2.99
6	2.68	3.13	18	2.21	2.68	30	2.19	2.56
7	2.78	3.21	19	2.29	2.77	31	2.43	2.87
8	2.39	2.73	20	2.15	2.54	32	2.47	2.68
9	2.74	3.09	21	2.64	3.29	33	2.81	3.24
10	2.41	2.73	22	2.16	2.70	34	2.68	2.75
11	2.47	2.65	23	2.54	3.26	35	2.39	2.99
12	2.61	2.59	24	2.24	2.74	36	2.47	2.94

**Table 4:** Comparison of the language test between the experimental group and the control group.

Number	PCS group	Control group	Number	PCS group	Control group	Number	PCS group	Control group
1	2.03	3.10	13	1.94	3.08	25	1.96	2.63
2	1.97	3.02	14	1.98	2.69	26	2.02	3.20
3	2.01	2.62	15	2.02	2.71	27	2.03	3.01
4	2.07	2.73	16	2.05	2.80	28	1.96	2.93
5	1.96	2.90	17	2.06	2.67	29	1.94	2.69
6	2.01	2.75	18	2.04	3.18	30	1.99	2.65
7	2.05	2.84	19	2.06	3.13	31	1.96	2.95
8	2.02	2.71	20	1.99	2.71	32	1.99	2.84
9	2.02	3.10	21	2.04	2.95	33	2.06	2.77
10	2.03	2.68	22	2.02	2.79	34	2.05	2.59
11	1.94	2.60	23	1.95	2.76	35	1.96	2.68
12	2.01	2.88	24	1.98	2.92	36	1.95	2.79

**Table 5:** Comparison of the visual space and executive function test between the experimental group and the control group.

Number	PCS group	Control group	Number	PCS group	Control group	Number	PCS group	Control group
1	2.37	2.72	13	3.19	2.90	25	3.23	2.96
2	4.16	2.86	14	2.96	3.20	26	3.42	2.89
3	2.38	3.12	15	3.46	3.10	27	2.73	3.13
4	4.27	3.14	16	4.20	3.16	28	2.44	2.92
5	3.99	2.98	17	3.12	3.02	29	3.98	3.06
6	2.64	2.79	18	2.67	3.14	30	2.56	2.84
7	2.51	3.01	19	4.01	3.12	31	2.64	2.93
8	3.40	2.76	20	4.31	2.83	32	4.37	3.00
9	2.46	3.01	21	3.21	2.94	33	3.22	2.96
10	4.57	2.91	22	4.63	2.94	34	3.77	3.09
11	4.02	2.93	23	3.44	2.83	35	3.58	2.68
12	3.68	3.13	24	3.64	2.96	36	3.78	2.75

**Table 6:** Comparison of the abstract test between the experimental group and the control group.

Number	PCS group	Control group	Number	PCS group	Control group	Number	PCS group	Control group
1	0.82	0.61	13	0.90	0.58	25	0.65	1.24
2	0.60	0.58	14	0.79	0.89	26	0.60	1.06
3	0.68	1.31	15	0.86	0.96	27	0.81	0.73
4	0.94	1.12	16	0.58	0.84	28	0.54	0.64
5	0.73	0.74	17	0.60	0.91	29	0.63	0.64
6	0.64	1.28	18	0.91	1.40	30	0.71	0.90
7	0.72	0.74	19	0.95	0.99	31	0.58	0.87
8	0.57	0.97	20	0.92	1.08	32	0.93	1.41
9	0.69	0.66	21	0.57	0.87	33	0.72	0.66
10	0.72	0.70	22	0.57	1.09	34	0.80	1.35
11	0.91	0.92	23	0.63	1.23	35	0.69	1.02
12	0.86	1.23	24	0.81	1.14	36	0.50	1.15

**Table 7:** Comparison of the delayed memory test between the experimental group and control group.

Number	PCS group	Control group	Number	PCS group	Control group	Number	PCS group	Control group
1	2.92	2.56	13	2.87	3.61	25	4.55	2.55
2	4.89	3.07	14	5.03	3.34	26	2.42	2.60
3	5.30	3.13	15	5.15	3.66	27	4.26	2.69
4	3.50	3.28	16	3.12	3.51	28	4.06	3.34
5	4.91	3.00	17	2.75	2.37	29	3.43	3.19
6	3.34	3.26	18	3.34	3.08	30	5.01	3.14
7	2.37	3.63	19	4.22	3.35	31	4.44	3.39
8	5.08	2.62	20	4.73	3.10	32	3.60	2.99
9	2.96	2.51	21	4.46	3.62	33	4.53	2.82
10	5.10	2.79	22	3.03	2.48	34	3.42	2.37
11	4.77	3.44	23	4.38	2.82	35	4.14	3.19
12	3.02	2.71	24	3.90	2.61	36	3.67	2.67

**Table 8:** The functionally connected brain regions with ROI on the left medial prefrontal lobe.

Brain area	Voxel value	*t* value
Fusiform gyrus	77	3.879
Putamen	131	-3.093
Putamen	79	-3.182
Superior temporal gyrus	73	2.790
Para hippocampus	40	3.906
Island leaves	68	-2.862
Subfrontal gyrus	65	-3.384
Subfrontal gyrus	63	-4.184
Middle temporal gyrus	98	2.287
Middle temporal gyrus	93	-2.959
Inferior forehead triangle	120	-3.141
Middle back	197	-4.070
Inferior forehead triangle	63	-2.746
Angular gyrus (lower apical leaflet)	60	-2.131
Medial superior frontal gyrus	65	-3.721
Top leaflet	71	4.442

**Table 9:** The functionally connected brain regions with ROI on the right medial prefrontal lobe.

Brain area	Voxel value	*t* value
Para hippocampus	33	3.976
Inferior temporal gyrus	51	3.594
Talar gyrus	125	-3.595
Apical leaflet	65	-2.746
Apical leaflet	47	-2.950
Central front back	90	-3.422
Central back	49	-4.356

## Data Availability

The data used to support the findings of this study are included within the article.
